This article has been retracted.

# The Effect of Tedlar Bags on the Composition of Exhaled Human Breath Samples

**DOI:** 10.1155/2022/5665921

**Published:** 2022-09-30

**Authors:** Jiuyan Zhao, Lanlan Zhu, Wei Zhang

**Affiliations:** ^1^Emergency Department, Guizhou Province, The Affiliated Hospital of Guizhou Medical University, No. 28, Guiyijie Road, Liuguangmen, Guiyang City 550004, China; ^2^Department of Respiratory and Critical Care Medicine, First Affiliated Hospital of Nanchang University, Nanchang University, Yong Wai Zheng Jie No. 17, Nanchang 330006, China

## Abstract

The PVF Tedlar is widely used for gas collection in clinical diagnostics and environmental research. However, sample collection is frequently associated with the degradation, adsorption, or transformation of sensitive chemicals. Here, we explore to what extent the Tedlar bag collection effects the composition of expired breath samples. Collected breath samples were analyzed using the EESI-MS technique after the storage time of 30 min, 1 h, 2 h, 3 h, 4 h, 5 h, and 6 h, respectively. Our results demonstrated the gradual MS signal decay after 3 h storage. The decay rate of 3 h is about 45% and 6 h is about 88%. Therefore, the Tedlar bag is suggested as a reliable breath holder on the time scale of <3 h.

## 1. Introduction

In recent years, exhaled breath and environmental air samples are popular samples for quality of life [1, 2]. These studies must collect sample gas with a standard method and with some commercial tools because of difficulty to collect representative sample gas reproducibly. An air-holding method is used to figure out the essential component of exhaled breath [3]. At present, sampling has been normally grabbed with the following tools: cylindrical acrylic chamber, air pump, and Tedlar bags [4–6]. Bags are often used rather than canisters. Firstly, bags are portable and easy to transport. Secondly, bags can be made from a series of materials, such as Tedlar, Teflon, foil, and Melinex sampling bags. Tedlar bags made from PVF (polyvinyl fluoride) film have been widely applied in several fields due to their adsorbing organic compounds, especially industrial hygiene, medical research, and environmental studies [7–9]. Many scientists are worried that Tedlar sampling bags do damage to the integrity of components, both odor and chemical. Still, the bags remain popular for their advantages [10]. Parker et al. [11] found that there was association between the intensity of odor and the laboratory DTFCO measurements and reported that the background of DTs in the Tedlar bags can be reduced to an acceptable level after heat-treating at 100°C. Beauchamp et al. [12]. showed that online PTR-MS (proton-transfer-reaction mass spectrometry) makes bag cleanliness for breath-gas sampling acceptable. Steeghs et al. reported that the use of laser-based photoacoustic detection results in less than 10% losses from exhaled breath samples (52 h after filling) and no significant reduction of ethylene over three days [13]. However, these primary literature reports do not address exhaled breath samples.

We observed the change pattern of exhaled air at 6 hours in the bag. The new platform, named EESI-ITMS (extractive electrospray ionization ion trap mass spectrometry) using a home-made EESI ion source coupled to a commercial LTQ (linear trap quadrupole) mass spectrometer [14, 15], was applied for exhaled breath analysis [16]. Under the optimized conditions, metabolic changes of humans were traced [17]. We have detected the components in the Tedlar bag changing with time using EESI-MS when these bags with N_2_ (99.999%) and exhaled breath, respectively. This study provides nonproprietary and essential information about the attenuation of exhaled breath and other gas with Tedlar bags.

## 2. Materials and Methods

### 2.1. Materials and Reagents

An LTQ-XL mass spectrometer (Finnigan, San Jose, CA, USA) with a home-made EESI ion source was employed in the experiment. The gas and exhaled breath samples were prepared with PVF bags (Dalian Delin Gas Packing Co., Ltd., Dalian, China) were cleaned consecutively 3 times with high-pure (99.999%) N_2_ and heated in the oven at 50°C for 30 minutes. All of the 5 L bags employed in this work were made of a single polypropylene fitting with integrated septum. Nitrogen (99.999%) (Tokyo Chemical Industry Co., Ltd., Tokyo) and HPLC-grade methanol (ROE Company, USA) were purchased. Ultrapure water with a resistivity of 18.2 MΩ/cm was supplied by a commercial water purification system (Barnstead Nanopure Ultrapure, Thermo Scientific, USA). A rotameter controlling the flow rate of exhaled breath was bought locally (Shenyang Zhengxing Flow Meter Co., Ltd., Shenyang, China). The PFA tube for the exhaled breath was replaced by a PTFE (Teflon/polytetrafluoroethylene) tube (ID 2 mm, OD 4 mm, Qiwei Industrial Material Co., Ltd., Dongguan, China).

### 2.2. Instrumentation and Working Conditions

The experimental setup has been described previously [18]; here, only a concise description is presented. The experimental setup is shown in Figure 1. The ESI high voltage was set at 3.5 kV, the temperature of the ion entrance capillary 100°C, and the pressure of the high purity nitrogen gas 1.2 MPa. The ESI solvent and the sample spray with 100% methanol were injected at a rate of 5 *μ*L min^−1^. 5 mm was set between the two spray channels of the EESI source (a) and 1-2 mm between the tips of the EESI source and the MS inlet (b). The angle between the two spray channels and the angle between individual sprays and the MS inlet were around 60° (*α*) and 150° (*β*), respectively. The flow rate of sample gas was 800 mL·min^−1^.

EESI-MS was used to test exhaled breath in the same optimized conditions as the nitrogen experiments (Figure 1). Ten Tedlar bags were filled with exhaled breath from a healthy volunteer with the same method, and the same storage conditions and were detected immediately and at 30 minutes, 1 h, 2 h, 3 h, 4 h, 5 h, and 6 h, respectively.

### 2.3. Data Analysis

The data were analyzed using Origin 9 software. The visible trend of curves was manually checked and separately confirmed by 2 independent reviewers.

## 3. Results

### 3.1. Experiment

Figures 2 and 3 show the nitrogen samples of directly detected and the 3 h nitrogen sample in (a) and (b) for positive and negative mode. From Figure 2, we can detect the most substance of signal after 3 h in Tedlar bags, for example, *m*/*z* 88, 197 and *m*/*z* 388 in Figure 2(a), and we can detect *m*/*z* 88, 197, 388 in Figure 2(b). Likewise, from Figure 3, we can detect the most substance of signal after 3 h in Tedlar bags, for example, *m*/*z* 88, 197 and *m*/*z* 388 in Figure 3(a), and we can detect the three substances in Figure 3(b). Comparing Figures 2 and 3, we have not found new generated substance after 3 h in Tedlar bags in a similar way.

### 3.2. Experiment

This study aims to test exhaled breath signal in Tedlar bags over time. We measured the signal of exhaled breath in the bags after 30 min, 1 h, 2 h, 3 h, 4 h, 5 h, and 6 h, respectively, and compared the signals.

In this study, Figure 4 shows the mass spectra of exhaled breath detected immediately and at 30 min, 3 h, and 6 h in EESI-MS. The *m*/*z* 279 and 301 signals are the biomarkers for exhaled breath. Apart from *m*/*z* 88, both signal intensity and peak density in the mass spectrum changed after storage in Tedlar bags for some time. For instance, intensity levels decreased dramatically among peaks including *m*/*z* 205, 279, and 301 stored in Tedlar bags (Figure 4). The enlarged view of the peak density was stored in 30 minutes (Figure 4(b)) within the mass range of *m*/*z* 50–400, and Figure 4(a) shows slight changes. The peak density stored in 6 h (Figure 4(d)) is much lower than that stored in 3 h (Figure 4(c)). These changes (from Figures 4(a) and 4(b)) of peaks are more obvious than those changes (from Figures 4(c) and 4(d)). On the other hand, before and after storage in Tedlar bags, it has little impact on the intensities for some peaks such as *m*/*z* 88 from Figures 4(a)–4(d). We observed that the signal of the bags gradually decay with time, particularly in 3 h, and the signal is less changed after 6 h.

In order to observe the variety patterns of mass spectrum peak, we record these mass spectrum peaks and draw graphics as shown in Figure 5. Compared the change of mass spectrum peaks, m/z 310, 279, 205, 88 at different time including detected directly using EESI-MS, detected these peaks at 30 minutes, 3 h and 6 hours in the Tedlar bag.

Consequently, decay efficients of these mass spectrum peaks were evaluated by this figure:

(1) $$\begin{array}{c} e_{3h}\approx 30\%-40\%,e_{6h}\approx 40\%-60\%. \end{array}$$

Compared the change of detected directly using EESI-MS and detected these peaks at 30 minutes in the Tedlar bag, the peaks of detection at 30 minutes are higher than the peak of direct detection, and the answer is probably that the density of these VOCs are relatively higher.

In Figure 5, the peak of *m*/*z* 88 does not decrease with time in the Tedlar bag. It has been found that *m*/*z* 88 is acetonitrile by the table of ESI + common background ions. The noble gases could not escape, and chemically unreactive gases such as acetonitrile would remain in the Tedlar bag.

## 4. Discussion

In this research, we analyzed the N_2_ and exhaled breath stored in Tedlar bags using EESI-MS detection. It has recently been shown that absorptive losses of VOCs (volatile organic compounds) were slower and less significant [19, 20]. It is more rigorous compared with previous studies of our project design and the process of collecting exhaled breath. Our results support the theory that absorptive losses are slight in Tedlar bags during the filling of acetonitrile. The results of our experiment are in general agreement with previous bag film studies in VOC testing and storage [21, 22]. We found that Tedlar bags are good for volatile gases and clean well. Tedlar bags can absorb components of exhaled breath and the signal of exhaled breath gradually attenuate with time, especially after 3 h. The decay rate of 3 h is about 35% and 6 h is about 50%. Therefore, it is concluded that exhaled breath can be more susceptible to negative bias than acetonitrile. Hence, we must test exhaled breath in the Tedlar bag quickly. It would be best to test the sample within three hours after sampling. Therefore, this evaluation of the Tedlar bag supports the use of Tedlar bags for exhaled breath to minimize the deviation between laboratories.

Compared with other studies [23, 24], we mainly study exhaled breath and analyze exhaled breath with more advanced mass spectrometer, so the results of the study are more accurate. Tedlar bags can be used to store exhaled breath for analysis and study. For these reasons, this study provides a time frame for researchers who need to use polyfluoroethylene bags.

Our study still has several limitations that should be concerned before a definite conclusion. Only one type of Tedlar bag was employed in this study without appropriate control bags. Therefore, Tedlar bags with different materials from different manufacturers should be applied as controls to draw a more solid conclusion in the future study.

## Figures and Tables

**Figure 1:** Schematic diagram of an EESI source.

**Figure 2:** EESI-MS spectrum of nitrogen in positive. (a) Detected directly, without bags. (b) 3 h in Tedlar bag.

**Figure 3:** EESI-MS spectrum of nitrogen in negative. (a) Detected directly, without bags. (b) 3 h in Tedlar bag.

**Figure 4:** Mass spectral fingerprints recorded from exhaled breath of the same volunteer using EESI-MS. (a) Detected immediately using EESI-MS. (b) 30 min in Tedlar bag. (c) 3 h in Tedlar bag. (d) 6 h in Tedlar bag.

**Figure 5:** The signal of VOCs gradually reduces with the increase of experimental time. *m*/*z* 301, 279, 205, and 88.

## Data Availability

The data used to support the findings of this study are included within the article.
